The article "An Empirical Analysis of Corporate Financial Management Risk Prediction Based on Associative Memory Neural Network" was published in 2021. Journal: Comput Intell Neurosci.

# An Empirical Analysis of Corporate Financial Management Risk Prediction Based on Associative Memory Neural Network

**DOI:** 10.1155/2021/4383742

**Published:** 2021-12-02

**Authors:** Hui Chu

**Affiliations:** China University of Mining and Technology-Beijing, School of Management, Beijing 100083, China

## Abstract

As a human brain-like computational model that can reflect the cognitive function of the brain, the problem of dynamic analysis of associative memory neural networks has attracted the attention of scholars. This paper combines associative memory neural networks with enterprise financial management risks, studies the synchronization control and stability analysis problems of unidirectional associative memory-like human brain amnestic neural networks with perturbation and mixed time-varying time lags, proposes a bidirectional associative memory-like brain stochastic amnestic neural network model with mixed time-varying time lags, designs a discrete-time sampling control strategy based on the model, and studies various types of recent financial risks. Based on the early warning research, based on the associative memory neural network method, we propose to reconstruct the risk categories, including improving the enterprise risk management system, enhancing the awareness of financial risk management from top to bottom, and strengthening the core competitiveness of the enterprise itself and control measures for financing, investment, operation, and cash flow risks.

## 1. Introduction

Associative memory neural network is by imitating the working pattern of neuronal cells in the human brain; firstly, the pattern to be memorized is stored in the form of weight network of the neural network; when receiving the information of incomplete or defective pattern from outside, the neural network at this time makes the input pattern continuously change its value and converge to the memorized pattern by massive parallel computation. The neural network has a good robust performance, which means that the associative memory neural network has a good fault tolerance performance. The patterns to be memorized are first stored in the form of a network of weights of the neural network. When receiving information about incomplete or fragmented patterns from outside, the neural network then continuously changes its values and converges to the memorized patterns through massive parallel computation. Associative memory neural networks are now widely used in pattern recognition, image processing, etc. Self-associative memory means that the input aberration patterns are equal to the remembered patterns; in contrast to heteroassociative memory, the input aberration patterns are not the same as the remembered patterns but show corresponding mapping relationships. Self-associative memory refers to the application of associative memory in which the initial pattern of input is identical to the remembered pattern of output. The first step in self-associative memory is to deposit the desired memorized pattern (e.g., the word computer) in a specific form into the network weights through the learning algorithm of a neural network [1]. Then, it is possible to input the pattern with cue information, and the neural network performs continuous iterative operations to give the correct output, and this cue information is not the complete word but has noisy information, but the neural network is still able to calculate to get the remembered word information; i.e., this associative memory neural network has a certain degree of fault tolerance. In fact, fault tolerance is one of the criteria to judge whether the application of associative memory is feasible. The memory process of the neural network, that is, the setting of the weights of the neural network, needs to translate the memorized patterns into the form of the state values of each neuron when the neural network is in a stable state; that is, generally, a stable point of the neural network can store a pattern, and the determination of the value of the stable point needs to be set according to the necessary conditions required by the associative memory neural network model adopted in this chapter, generally by substituting the memory pattern into the set of differential equations of the neural network, then listing the corresponding inequality based on the above necessary conditions, and relating this inequality to the system of differential equations coupled to solve a specific set of solutions and eventually determine a more suitable weight [2]. This process is also performed using specific training algorithms (e.g., through network self-feedback). Since the self-associative memory input and output patterns are identical, meaning that both have the same dimensionality, this is a characteristic of self-associative memory.

The article "An Empirical Analysis of Corporate Financial Management Risk Prediction Based on Associative Memory Neural Network" was published in 2021. Journal: Comput Intell Neurosci.

Under the conditions of market economy, enterprises must be aware of the objectivity of financial risks, and at present, enterprises generally have a weak awareness of financial risks, blind fund-raising, imprudent investment, inadequate financial risk management system, and state-owned enterprises, which have weak points such as imperfect financial risk evaluation mechanism and lack of risk control measures. Thus, studying the characteristics of enterprise financial risks and taking certain measures to prevent and manage them has become an important issue facing us now. Although the rapid development of various industries also brings many risks, the industry frequently appears in the financial crisis and even eventually leads to bankruptcy of enterprises [3]. The determination of the stability point value is set according to the necessary conditions required by the associative memory neural network model adopted in this chapter, generally by substituting the memory model into the set of differential equations of the neural network and then listing the corresponding inequalities according to the above necessary conditions. This inequality is then combined with the set of differential equations to solve a series of specific solutions and finally determine a more suitable weight value. Therefore, the financial risk management of enterprises is very important and can determine whether the enterprise can develop in a high speed and sound manner. In recent years, scholars have also increased their research on the financial risk management of enterprises, but a systematic theoretical system has not yet been formed for the study of the financial risk of enterprises. Furthermore, the focus of existing research is to analyze the financial risks of enterprises and put forward financial risk control opinions, and there are relatively few studies that analyze the steps of financial risk management of enterprises, i.e., the identification, evaluation, and control means of financial risks, in-depth. Based on associative memory neural network, this paper combines the relevant theoretical literature on enterprise financial risk control with the specific case of financial risk control of the Storm Group and researches the identification, analysis, and evaluation of financial risk and control of enterprises, hoping to play a supplementary verification role to the current theoretical research on financial risk control in enterprises.

## 2. Status of Research

Artificial neural networks have been intensively studied in recent decades due to their wide application in many fields such as pattern recognition, associative memory, signal processing, and optimization. Some applications, such as those in optimization theory, require neural networks to have only a single stable point. However, some other applications such as associative memory and pattern recognition require the existence of multiple stable equilibria in the neural network itself.

The multistability of two recurrent neural networks with phase plane origin symmetric activation functions is studied in the literature [4]. Multiple *μ*-stability of neural networks with unbounded time-varying time lags is considered in the literature [5]. The multistability of recurrent neural networks with nonmonotonic activation functions and unbounded time-varying time lags is discussed in the literature [6]. In the literature [7], the multistability of fractional-order neural networks in the Mittag-Leffler sense with segmental constant parameters is discussed. The multistability of a class of Hopfield neural networks with stochastic time lags was studied in the literature [8] by applying Schauder's immobility point principle and the related stochastic time-lag theory, where there exist 2*n* rectangular invariant set regions under certain conditions and at least one of these regions has an equilibrium point, and by proposing two sufficient conditions to ensure that these equilibrium points are stable. A new condition that is less restrictive relative to the Lipschitz continuum condition in complex-valued activation functions is proposed in the literature [9], and a series of criteria are presented to guarantee the existence, uniqueness, and numerical examples of global asymptotic stabilization points of complex-valued recurrent neural networks. In the literature [10], the stability of recurrent neural networks with time-varying time lags is analyzed using FTM (Flexible Edge Method), and several new stability criteria are proposed to describe the stability of this neural network by constructing a new type of Lyapunov function. In the literature [11], a novel design idea for CVHAMs (complex-valued multistate Hopfield associative memory) is proposed to analyze the stability of CVHAM systems utilizing the energy function method and finally obtain that the network can converge to an immobile point for an arbitrary input value, and the projection geometry of the GPR (generalized projection rule) is discussed. According to the literature [12], Internet enterprises have the financial characteristics of the “flow economy” model, asset-light operation model, cost-light and expense-light, fast product replacement, and equity financing. The financial risk of Internet enterprises has both the characteristics of general enterprises and its special characteristics. Compared to the general enterprises, the risk of capital shortage of Internet enterprises is the most significant. The literature [13] introduced the EVA valuation model to explore the link between financial risk and an enterprise value of Internet enterprises, used the EVA model and the traditional valuation model to assess the company value of the case company NetEase, and concluded that the EVA valuation model is more accurate. The literature [14] argues that Internet enterprises mainly have risks in profitability model, cash flow, financing, investment, and government regulation. It also suggested that Internet enterprises should establish a sound financial risk early warning mechanism, set up a professional auditing institution and audit system, strengthen comprehensive budget work, improve the accounts receivable control mechanism, and strengthen financing and investment risk management. The literature [15] argues that the assurance of asset profitability and the control measures proposed to prevent unexpected losses are accomplished through risk management. Literature [16] argues that companies should first establish a sound internal control system when making business decisions, which can, to a certain extent, avoid suffering financial risks and causing operational difficulties when financing activities. Literature [17] studies the origin of the risk, the financial risk mechanism of action as the goal to explore, and more targeted risk identification, evaluation, and control, eliminating the hidden financial risk factors.

The article "An Empirical Analysis of Corporate Financial Management Risk Prediction Based on Associative Memory Neural Network" was published in 2021. Journal: Comput Intell Neurosci.

## 3. A Risk Model for Corporate Financial Management Based on Associative Memory Neural Networks

### 3.1. Associative Memory Neural Network Model

The basic steps of the current recurrent neural network training algorithm are to first preprocess the samples to be recognized to obtain numerical feature vectors, input these vectors sequentially into the network, then compare the output of the network with the going output by a difference, and use this difference as negative feedback to correct the network weights. The advantage of this algorithm is that it is simple to operate and the training process is unsupervised learning, while the disadvantage is also evident in that it needs to be retrained once every time a new sample pattern is remembered, which may consume more time in the case of larger network dimensions. The neural network model is built by adjusting the weights of its neurons after it receives data, and the input variables of the model can change according to the actual needs, such as market factors and financial indicators. The neural network model can be automatically trained to filter the best variables and adjust the weights according to their implied relationships to build a nonlinear model and improve the model accuracy. The training method is used to correct the network weights by continuously feeding in training samples so that the sample patterns to be remembered are embedded in the network weights; i.e., the network “remembers” the samples. It is possible to use algebraic methods to solve the weights directly, because the network has a large number of attractors and can remember a large number of samples, by using the samples as input, assuming that the output is the desired output, representing both as vectors, and substituting them into the differential equations of the system, using the knowledge of linear algebra to solve a set of weights network, then using other samples for input, and finally solving the corresponding number of analytical solutions. The intersection of these analytic solutions is the network of weights to be determined if these solutions do not intersect. Then, it means that the memory capacity of the network is not sufficient and a new model needs to be redesigned to ensure that it has sufficient memory capacity [18]. Next, an example of the design of associative memory will be given, as shown in Figure 1 for an example of the associative memory process.

The article "An Empirical Analysis of Corporate Financial Management Risk Prediction Based on Associative Memory Neural Network" was published in 2021. Journal: Comput Intell Neurosci.

Here is an example of the detailed steps of associative memory design; a recurrent neural network can be described by the following set of differential equations:

(1) $$\begin{array}{c} \frac{\partial }{\partial W_{ij}^{l}}J\left(w,b\right)=\frac{1}{b}\sum_{i=1}^{m}J\left(w,b;x^{i},y^{i}\right)+\lambda W_{ij}^{l}. \end{array}$$

The network is a more classical model of a memetic recurrent neural network. Several character samples are used for the training of this network until the network is given a network of weights that satisfy the conditions that make the network remember the characters to be remembered. For the sample image data to be recognized, the image first needs to be subjected to a series of preprocessing steps, which are graying, smoothing, denoising, and finally, transforming into an input vector. All samples of data are grayed out, smoothed, denoised, and then transformed into an array of vectors of the following form:

(2) $$\begin{array}{c} f_{\phi }\left(p,x\right)=d_{p}\left(x-\frac{\lambda_{\theta_{1}}}{d_{p}\left(x\right)}\right)+d_{p}\left(x-\frac{\lambda_{\theta_{2}}}{d_{p}\left(x\right)}\right). \end{array}$$

And the output vector of the network can be represented as an array of vectors of the form

(3) $$\begin{array}{c} \left(\alpha ,\beta ,\gamma \right)=\frac{1}{r}\sum_{i=1}^{k}\left(\frac{\alpha_{i}+\beta_{i}+\gamma_{i}}{3}\right). \end{array}$$

Substituting the above two sets of vectors into the system equation (1), we get

(4) $$\begin{array}{c} \nabla_{b^{t}}J\left(w,b;x_{i}^{*},y\right)=\delta^{l+1}\frac{\partial J\left(w,b\right)}{\partial b_{ij}^{l}}+\lambda \alpha_{ij}^{l}, \end{array}$$

where *x*_*i*_^*∗*^*x*_i_∗ is the stable equilibrium point of the system with the *i*-th set of samples as input, and this value is chosen according to conditions such as the form of the activation function. A sufficient condition for this equation to have a solution is that the number of stable equilibrium points of the neural network is greater than or equal to the number of samples to be memorized by the claim; that is, the number of attractors should be large enough to be able to remember a sufficient number of patterns. The equation can be solved using singular value decomposition, the solution of the equation is also the vector of connection weights of the network, and these weights imply information about the patterns to be remembered. The above form is generally a self-associative memory weight solving process that can be specifically applied in the fields of character recognition, face recognition, etc. Then examples will be given to illustrate the design and the weight solving process of recurrent neural network-based heteroassociative memory applications. Traditional character recognition algorithms include template matching and OCR [19]. For unbalanced sample data, you can start with downsampling and upsampling methods. The downsampling method, also known as the random downsampling method, refers to the random removal of the class of data with the most categories by the sampling method. The advantage is that the sampling method can improve the model accuracy when the deleted samples contain noisy data, and the disadvantage is that some important samples may be deleted. Oversampling method refers to synthesizing a part of small sample data by an algorithm. Compared with these character recognition algorithms, the recurrent neural network-based associative memory mentioned above is characterized by low design cost, simple processing logic, fast network convergence, less dependence on external conditions, and easy practical implementation. The most important point is that this associative memory system has good fault tolerance performance; high fault tolerance means that when there is more noise or disturbance in the sample, it can also correctly identify the target pattern, so if this associative memory method is applied to image recognition, although the current application is simple and the idea is more basic, after a little development, I believe there will be a use for it. The design steps of recurrent neural networks for associative memory are summarized as follows.

1. Determine the model characteristics of the neural network to be used
2. Convert the patterns to be remembered into vectors as inputs to the system as well as outputs to be substituted into the system equations
3. The solution to the system of equations is obtained by appropriate choice of coordinates of the equilibrium point and by singular value decomposition
4. Store the solutions of the system of equations as the weights of the neural network
5. Build an associative memory neural network system and perform recognition tests.

The article "An Empirical Analysis of Corporate Financial Management Risk Prediction Based on Associative Memory Neural Network" was published in 2021. Journal: Comput Intell Neurosci.

The associative memory-based reconfigurable amnestic network circuit consists of four parts: the associative memory-based amnestic network circuit, the PRMC with input binary signals, the synaptic circuit block, and the control circuit. In the associative memory-based amnestic network circuit, the synaptic weights indicate the strength of the synaptic connections and thus only positive weights. The PRMC of the input binary signal can only be trained by the algorithm to achieve the corresponding function, so the synaptic circuit needs to represent negative weights, zero weights, and positive weights. In the associative memory-based reconfigurable memetic neural network circuit, the PRMC with input binary signals and the associative memory-based memetic neural network circuit uses the same synaptic circuit, and the synaptic circuit in the associative memory-based memetic neural network circuit is restricted to vary within the positive weights by a control circuit [20]. The synaptic circuits in the synaptic circuit block are shared, and these synaptic circuits can be used to construct both PRMCs with input binary signals and the associative memory-based memetic neural network circuits. As can be seen in Figure 2, the two subnetworks operate independently, so they can work in parallel.

By simulating learning and forgetting in associative memory, the reconfigurable memristor neural network circuit based on associative memory can dynamically change the circuit structure to achieve reconfiguration, corresponding to the following process: when the unconditioned stimulus signal and the conditioned stimulus signal are simultaneously input to the memristor neural network circuit based on associative memory, associative learning between the two is induced, so that the synaptic weight corresponding to the conditioned stimulus gradually increases. After the learning process is over, if the conditioned stimulus signal is kept input, the forgetting process is induced. During forgetting, the synaptic weight corresponding to the conditioned stimulus gradually decreases until it fails to activate the corresponding neuronal circuit. After the end of the forgetting process, the circuits of the associative memory-based amnestic network do not activate regardless of whether the conditioned stimulus signal is input [21]. And then, the synaptic circuits corresponding to the conditioned stimulus can be disconnected from the neuronal circuits, and these synaptic circuits can be fed into the synaptic circuit block. The synaptic circuits in the synaptic circuit block can be used to construct either PRMC or associative memory-based amnestic network circuits with input binary signals. In this way, circuit reconfiguration is achieved.

The article "An Empirical Analysis of Corporate Financial Management Risk Prediction Based on Associative Memory Neural Network" was published in 2021. Journal: Comput Intell Neurosci.

## 4. An Associative Memory Neural Network-Based Risk Prediction Model for Corporate Financial Management

Financial risk is a type of business risk that exists in financial activities such as raising, investing, spending, recovering, and allocating activities of funds in the process of social reproduction. And the risk is the deviation of expectations from reality. There is a distinction between financial risk in a narrow and broad sense. Financial risk in the narrow sense refers to the financial risk arising from the debt operation in the process of raising funds for the enterprise. Financial risk in the broad sense refers to the uncertainty of obtaining the expected financial results in the process of conducting the financial activities of the enterprise. Therefore, the financial risk exists in every enterprise and in the business activities of the enterprise and has a significant impact on the profit and loss situation and business conditions of the enterprise. Financial risk management is the prevention, control, and management of risk in enterprise financial management and is also a part of comprehensive enterprise risk management [22]. Internal diagnosis is a way for the enterprise itself to find out various problems in the business process through self-analysis and finally to solve them in a targeted manner. External diagnosis means that the enterprise hires an external third-party organization to analyze the financial operation of the enterprise. As a new management science theory, it is a management theory mainly developed by scholars according to the previous experience in risk management and financial management for all kinds of risks in the operation of enterprises. Financial risk management includes risk identification, assessment, analysis of causes, and control of various financial activities of the enterprise. To ensure the normal operation and capital movement of the enterprise and to avoid negative impact on the economic interests of the enterprise, the management process of financial risk management includes risk identification, assessment, analysis of causes and control of various financial activities of the enterprise, and timely and effective prevention and control measures based on its early warning role.

The most commonly used methods for financial risk evaluation include hierarchical analysis, efficacy factor method, and factor analysis. The basic principle of factor analysis is to group indicators with strong relevance into one category and replace each category with a factor, thus replacing all the original indicators with a few factors.

The article "An Empirical Analysis of Corporate Financial Management Risk Prediction Based on Associative Memory Neural Network" was published in 2021. Journal: Comput Intell Neurosci.

In this paper, the analysis of corporate financial management risk prediction is carried out by combining the associative memory neural network model with factor analysis. Factor analysis is chosen for the following reasons: firstly, factor analysis can reduce the number of original variables, by extracting and naming the main factors instead of the vast majority of the original information; secondly, the sample can be ranked and compared. According to the score of each main factor and the comprehensive score, the sample can be ranked, which not only shows the ranking of individual factors and clarifies which factors have a greater impact on the financial situation of the enterprise but also analyzes the comprehensive ranking of the factors after weighting, which is beneficial to the enterprise to clarify its strengths and weaknesses [23].

The steps of the factor analysis method are as follows:

(1) KMO and Bartlett's test were performed to determine whether the original variables were suitable for factor analysis; KMO was used to describe the magnitude of the correlation coefficient between variables, and the larger the value, the more suitable for factor analysis; while the smaller the value of Bartlett's test, the more suitable for factor analysis.
(2) Constructing factor variables and extracting principal component factors in place of all initial variables, the mathematical model for factor analysis is
  (5) $$\begin{array}{c} f\left(\left\{x_{1},x_{2},\ldots ,x_{n}\right\}\right)=g\left(h\left(x_{1}\right)+h\left(x_{2}\right)+\cdots +h\left(x_{n}\right)\right). \end{array}$$
(3) Interpretation of the principal component factors is named, generally using the orthogonal rotation method to obtain the maximum loading values of the principal factors and clarify the meaning of what each factor represents.
(4) The expressions of each principal factor are derived from the component score matrix, and then a comprehensive evaluation model is constructed according to the respective weights, and the samples are ranked and analyzed.
  (6) $$\begin{array}{c} C_{ij}=\sum_{i=1}^{n}x_{i}^{2}\sigma_{i}+\sum_{j=1}^{n}x_{j}^{2}\sigma_{j}+\sum_{k=1}^{n}x_{k}^{2}\sigma_{k}. \end{array}$$

Associative memory neural network is built based on decision tree model using histogram algorithm which is easier to segregate the data. The difference from previous decision tree models is that the associative memory neural network is oriented vertically, i.e., generating the leaves of the decision tree, whereas other decision tree models generate the levels of the tree, so the associative memory neural network algorithm runs faster and stores fewer data. Its main feature is to traverse the entire training set and to make the attributes discrete for floating-point continuous variables; these *k* discrete data are constructed into a histogram with a specific width of *k*. The number of discrete values converged within each histogram is calculated. Since there are many components of financial risk, various factors and financial indicators will interact with each other to form a complex relationship. In this paper, relevant indicators are extracted, factors are extracted by significance test, and factors suitable for model building are obtained by sphericity test, principal component extraction, and other steps. Based on the obtained factors, the logistic model of stepwise regression is used to model the financial early warning. The modeling process gradually analyzes the factors of risk composition, using the advantages of the model to provide a more intuitive basis for the future decision-making of managers. The selected early warning indicators should be comprehensive; i.e., indicators should be selected from the traditional aspects of solvency, profitability, development capability, and operating capability, and indicators should be selected from the aspects of research and development capability that reflect the characteristics of the industry, making the range of indicators selected for the communication equipment manufacturing industry more comprehensive. The company invests capital in the production of products and recovers the capital and profits through the sales of the products. Inventory turnover can only be increased if sales are successful and inventory is cleared quickly, so inventory turnover indicates how quickly money can be recovered from the sale of goods. In general, a company can improve its liquidity by increasing its inventory turnover. The inventory turnover ratio indicates the level of inventory, while the current asset turnover ratio reflects the speed of turnover of current assets, which is the most liquid of all the assets of a company. A lower level of current asset turnover can have a greater impact on a firm's short-term repayment ability. The higher the current asset turnover ratio, the lower the relative financial liquidity risk. A slow turnover rate will require supplementary liquidity to participate in the turnover, which will create a waste of funds and reduce the profitability of the enterprise. Based on the above theory, in the subsequent classification, the optimal cut-off point can be found only according to the width of the histogram. The idea of the histogram algorithm is mainly reflected in the conversion of floating-point data into binary data, and the specific operation is to determine the number of buckets contained in each feature, update the data of each bucket separately after equal division, and substitute the features of enterprise financial management risk prediction into the associative memory neural network model, which is represented graphically as shown in Figure 3.

The article "An Empirical Analysis of Corporate Financial Management Risk Prediction Based on Associative Memory Neural Network" was published in 2021. Journal: Comput Intell Neurosci.

Compared to other models built on decision tree algorithms, associative memory neural networks are faster mainly in terms of running speed, while consuming less memory, and accuracy is not compromised, perfectly combining both fish and bear's paw. With the desire to go to the next level, the model can be optimized in the following two ways: to speed up the running speed, the original data can be simply processed; reducing the number of features and data, converting feature variables into category features, or saving the data files as binary files, changing the training method of the model to parallel can also speed up the running speed of the model; to improve the accuracy of the model and reduce the model learning rate, starting from the model, mesh tuning the parameters of the model, choosing the best combination of parameters, increasing the learning times of the model, and making the model better understand the laws between the data can improve the accuracy of the model. Starting with the data, increasing the number of training data and preprocessing the data to solve the missing values and imbalance in the original data can also train the model better and improve the performance of the model.

### 4.1. Experimental Verification and Conclusions

The CART decision tree model with prepruning and postpruning design will be trained, and the decision tree graph and variable importance graph will be generated after the model training to better interpret the CART decision tree model discriminant results. Firstly, the discriminant results and ruleset of the overall financial risk assessment model of the enterprise are constructed. Because there are too many values of assessment features in the overall financial risk assessment of the enterprise, the variable importance graph in the overall financial risk assessment of the enterprise takes the top 5 importance variables, and the overall financial risk assessment model of the enterprise generates the variable importance graph as shown in Figure 4.

As can be seen from Figure 4, among the 18 characteristics of the CART decision tree model, “interest earned multiple,” “total assets return,” “accounts receivable turnover,” “total assets turnover,” and “weighted return on net assets” ranked the top five in importance, with “interest earned multiple” being the most important indicator with the importance of over 0.5. Operating capacity reflects the efficiency and effectiveness of an enterprise's capital operation with different assets, and the turnover efficiency of different types of assets is usually used to determine the operating level of an enterprise. This indicates that enterprises should focus on “interest earned multiple” when assessing the overall financial risk, and the sum of the top five importance scores exceeds 90%; therefore, it also indicates that listed companies should focus on these five index characteristics in the process of assessing the overall financial risk of enterprises. The interpretation of the rule set generated by the decision tree model will provide quantitative evidence for the listed company to assess the overall financial risk of the company, which will help the listed company to measure whether it has overall financial risk.

The article "An Empirical Analysis of Corporate Financial Management Risk Prediction Based on Associative Memory Neural Network" was published in 2021. Journal: Comput Intell Neurosci.

The importance of the variables generated by the enterprise operational risk assessment model is shown in Figure 5. As can be seen from Figure 5, the importance of the six characteristics of the CART decision tree model is the same, with the importance of “operating profit margin” becoming the most important assessment indicator. Therefore, the model results indicate that listed companies should focus on these 6 indicators in the process of enterprise business risk assessment. Rule 1: when the “operating profit margin” is ≤−6.151, the enterprise has business risks. Rule 2: when “operating profit margin” >−6.151 and “accounts receivable turnover ratio” >3.203, the company does not have financial risk. Rule 3: when “operating profit margin” >−6.151, “accounts receivable turnover” ≤3.203, and “cost margin” ≤7.552, the enterprise, there is financial risk. Rule 4: when “operating profit margin” >−6.151, “accounts receivable turnover” ≤3.203, and “cost margin” >7.552, the enterprise does not have financial risk. The interpretation of the rule set generated by the decision tree model will provide the listed company with quantitative evidence to assess the degree of the business risk of the company, which will help the listed company to measure whether it has business risk.

The importance diagram of the variables generated by the enterprise financing risk assessment model is shown in Figure 6. For the decision result of the CART decision tree model, among the three characteristics of financing risk, the importance of “interest multiples earned” becomes the most important evaluation indicator, and the importance score of its indicator is close to 0.8. Therefore, the model results indicate that listed companies should focus on the following characteristics in the process of enterprise financing risk evaluation. The year-over-year revenue growth rate, net asset per share growth rate, and total asset growth rate are important indicators of a company's growth ability. The model results suggest that listed companies should focus on the indicator characteristic of “interest multiples earned” in the process of corporate financing risk assessment. The set of rules for the determination of the CART decision tree for corporate financing risk is as follows. Rule 1: when the “interest earned multiple” is ≤1.249, the enterprise has financing risk. Rule 2: when the interest earned multiple is >1.249, the firm is not at risk. The interpretation of the rule set generated by the decision tree model will provide the listed company with quantitative evidence to assess the level of funding risk of the company, which will help the listed company to measure whether it has funding risk.

The article "An Empirical Analysis of Corporate Financial Management Risk Prediction Based on Associative Memory Neural Network" was published in 2021. Journal: Comput Intell Neurosci.

From Figure 7, it can be seen that this paper's model based on associative memory neural network achieves 83% accuracy for the discriminative effect of the training set and 76% accuracy for the validation set, which is a better result. At the same time, this paper combined the GBDT model with the logistic regression model for the combined prediction, and the prediction results showed that the combined model improved the prediction accuracy of the training set to 91% and the validation set to 78%, in terms of both accuracy and stability; the combined model warning effect is more significant compared with the single model, so it proves the feasibility of the combined model. Compared with the single model logistic regression model, the ROC curve of the associative memory neural network model regression financial risk warning model is closer to the upper left axis, and its AUC value is 0.79, which is significantly higher than the logistic regression model AUC value of 0.60. The advantages of the associative memory neural network financial risk warning model can be seen directly from the ROC curve and AUC value. From the experiment, it can be concluded that GBDT for feature combination can better mine the information in the financial data of listed companies, and the logistic model has fast processing speed, which can solve the problem of slow processing speed that GBDT cannot be processed in parallel, and the model fused with GBDT and logistic model can be effectively used in the field of financial risk early warning of listed companies for modeling.

The learning rate is the rate at which the input variables are updated at each iteration during training and determines how far the weights have to move in the direction of the gradient in a small batch, through many iterations, eventually moving to a position that matches the training accuracy of the network. The process of learning the features of a sample dataset by an associative memory neural network is the process of constantly iterating forward. A lower learning rate makes the training process more reliable, but optimization will take longer. Higher learning rates, on the other hand, lead to nonconvergence of training and may cause very large weight changes, making the loss function very poor. Optimizing the rate of matrix multiplication and improving memory utilization can be achieved by increasing the number of batches in a certain region, which reduces the number of updates needed to complete the training of the entire dataset and speeds up the process somewhat for data of the same capacity. Stochastic gradient descent updates only one sample information at a time, which speeds up the training, but because only one sample is used at a time, it does not represent the entire training sample, making it more difficult to converge the training results to some minimum value. For a company to achieve sustainable development, it must attach great importance to its R&D and innovation capabilities. Only through continuous innovation and continuous inventions can a company gain a competitive advantage. With the development of deep learning, it was shown that the training results could be converted to a local minimum by slowly decreasing the learning rate. After adjusting the parameters several times, the expected training results were finally obtained, and the average absolute error of the model on the samples during training finally converged. The loss curves for the sample dataset are shown in Figure 8.

The article "An Empirical Analysis of Corporate Financial Management Risk Prediction Based on Associative Memory Neural Network" was published in 2021. Journal: Comput Intell Neurosci.

The blue line in the figure represents the training set loss curve and the orange line represents the test set loss curve; the horizontal axis presents the number of iterations of the samples in the training process, and the vertical axis presents the change of the average error value during the training process. According to the parameters set in this paper, the Spyder window can display the losses of the training and test samples in each iteration and calculate the root mean square error of the model at the end of training. During the training process, the more iterations, the smaller the sampling error, with local fluctuations in a small range. At the beginning of the training, the error drops quickly, and in the training interval from 10 to 50 iterations, the error drops at a rapid rate, indicating that the model is being fine-tuned locally, and from 100 training iterations onwards, the error drops more gently, indicating that the model has converged to an optimal process. The trend of the loss curve of the training sample and the loss change of the test sample are integrated, and the error of the training sample finally converges with a better fit; the error of the test sample converges to a local minimum, and its fit is not as good as that of the training sample, but the effect of using gradient descent for optimization is obvious and will not affect the performance of the whole model.

The article "An Empirical Analysis of Corporate Financial Management Risk Prediction Based on Associative Memory Neural Network" was published in 2021. Journal: Comput Intell Neurosci.

Based on the associative memory neural network model, the early warning indicator system that can reflect the risk characteristics of listed agricultural companies is established by combining the risk characteristics of the company and the causes of its generation: it contains financial and nonfinancial indicators, covering solvency, operating capacity, development capacity, profitability, and other capacity indicators. To improve the convergence speed and stability of the model, SPSS software is used to conduct factor analysis on the data of the primary selected indicators and calculate the factor scores of the samples as the input layer data of the model. In this way, the accuracy of the financial crisis model is further determined and a part of the sample is selected to test the model. Finally, the model is applied to the actual company to identify its problems and optimize them to reduce the possibility of its financial crisis.

## 5. Conclusion

Associative memory neural network models are generally constructed based on data about the characteristics of the industry in question to make predictions about various aspects of demand points. Associative memory neural network model predictions are not only limited to daily life preferences, food, clothing, housing, etc. but now also almost permeate in financial industry development, financial forecasting, etc. In this paper, by analyzing the subsequent development capability in conjunction with the industry characteristics and competitive landscape of the company, it is found that the model can reflect the situation of the company well through early warning indicators and provide a reference for the future development of the company. If only the data model fitting of financial indicators is introduced, it will be too single and will not be able to judge the situation of finance comprehensively. In the study, it was found that the number of samples in the high financial risk category was too small compared to the samples in the low and medium financial risk categories, and if the sample data were not balanced, it might lead to the early warning model not learning the characteristics of the samples in the high financial risk category during training, which eventually led to a low prediction accuracy of the samples in this category. Since factors such as company composition and equity can also have an important impact on finance, this paper adds nonfinancial indicators to improve the generalizability and accuracy of the model. Nowadays, companies are in an increasingly complex market environment and social activities, and big data simulation by quantifying the relevant indicators of companies in the industry can reflect the current situation of the industry comprehensively and extensively, and the reasonable inclusion of industry-specific indicators can also improve the effectiveness of the early warning model. By combining the company indicators and the established early warning model, the principal components that can be identified by the model are used to analyze the situation in which the company risks arise while providing opinions that incorporate the details of Company B. Using this financial early warning model, one can adjust the company structure, do strategic planning and crisis prevention in advance for the changing market, organize training for financial early warning talent, strengthen the communication between financial early warning talents, and ensure a reasonable shareholding structure to avoid one share being dominant; secondly, one can improve the information construction of the financial system and establish a set of the financial system applicable to the company on this basis. At the same time, we should comply with the choice of the market, and the development of diversified markets can ensure their competition and at the same time focus on product quality.

The article "An Empirical Analysis of Corporate Financial Management Risk Prediction Based on Associative Memory Neural Network" was published in 2021. Journal: Comput Intell Neurosci.

## Figures and Tables

**Figure 1:** Example of the associative memory process.

**Figure 2:** Structural diagram of reconfigurable amnestic network circuit based on associative memory.

**Figure 3:** Flow chart of an interactive product styling model.

**Figure 4:** Importance of variables for assessing the overall financial risk of an enterprise.

**Figure 5:** Importance of business operational risk assessment variables.

**Figure 6:** Importance of variables generated by the enterprise financing risk assessment model.

**Figure 7:** Model accuracy validation.

**Figure 8:** Loss curve of sample size set for associative memory neural network.

## Data Availability

The data used to support the findings of this study are available from the corresponding author upon request.
